# Extravascular lung water index improves the diagnostic accuracy of lung injury in patients with shock

**DOI:** 10.1186/cc10599

**Published:** 2012-01-03

**Authors:** Michelle S Chew, Lilian Ihrman, Joachim During, Lill Bergenzaun, Anders Ersson, Johan Undén, Jörgen Ryden, Eva Åkerman, Marina Larsson

**Affiliations:** 1 Department of Intensive Care Medicine, Skåne University Hospital Malmö, Södra Förstadsgatan, Lund University, S-20502 Malmö, Sweden

**Keywords:** acute respiratory distress syndrome, acute lung injury, extravascular lung water, sepsis, shock, pulmonary oedema, likelihood ratio

## Abstract

**Introduction:**

The diagnosis of acute lung injury (ALI) may be more robust if more accurate physiological markers can be identified. Extravascular lung water (EVLW) is one possible marker, and it has been shown to correlate with respiratory function and mortality in patients with sepsis. Whether EVLW confers diagnostic value in a general population with shock, as well as which index performs best, is unclear. We investigated the diagnostic accuracy of various EVLW indices in patients with shock.

**Methods:**

We studied a prospective, observational cohort of 51 patients with shock admitted to a tertiary ICU. EVLW was measured within 6 hours of ICU admission and indexed to actual body weight (EVLW/ABW), predicted body weight (EVLW/PBW) and pulmonary blood volume (EVLW/PBV). The relationship of these indices to the diagnosis and severity of lung injury and ICU mortality were studied. Positive and negative likelihood ratios, pre- and posttest odds for diagnosis of lung injury and mortality were calculated.

**Results:**

All EVLW indices were higher among patients with lung injury and significantly correlated with respiratory parameters. Furthermore, all EVLW indices were significantly higher in nonsurvivors. The use of EVLW improves the posttest OR for the diagnosis of ALI, acute respiratory distress syndrome (ARDS) and severe lung injury (sLI) by up to eightfold. Combining increased EVLW and a diagnosis of ALI, ARDS or sLI increases the posttest odds of ICU mortality. EVLW/ABW and EVLW/PBV demonstrated the best diagnostic performance in this population.

**Conclusions:**

EVLW was associated with degree of lung injury and mortality, regardless of the index used, confirming that it may be used as a bedside indicator of disease severity. The use of EVLW as a bedside test conferred added diagnostic value for the identification of patients with lung injury.

## Introduction

Extravascular lung water (EVLW) is an estimation of the fluid in the pulmonary interstitial and alveolar spaces [1]. In ICUs, EVLW is usually obtained as one of the parameters in the PiCCO monitor (PiCCO *plus*; PULSION Medical Systems, Munich, Germany) by using a transpulmonary thermodilution technique. EVLW may be used as a bedside indicator of extravascular leakage, such as in a patient with acute lung injury (ALI) [1-7], although this requires further confirmation.

The present study was driven by current limitations in the diagnosis and prognosis of ALI and ARDS. For example, the North American-European Consensus Conference (NAECC) criteria may be too insensitive for identifying 'subclinical ARDS'. Conversely, their specificity has also been questioned because some patients identified by these criteria no longer fulfil the criteria for ARDS after 24 hours on mechanical ventilation [8]. Furthermore, it is known that the Lung Injury Score (LIS) and the ratio of partial pressure of oxygen in arterial blood to the fraction of inspired oxygen (PaO_2_/FiO_2_) lack sensitivity for predicting mortality [9], although they are clearly indicative of lung injury. It has been proposed that the diagnosis and prognosis of lung injury may be more robust if more accurate physiological markers can be identified. EVLW has been proposed as one such method [10-12], and there are a number of studies attesting to the value of EVLW for clinical outcome prediction [2,4,5,13-17].

In previous studies, EVLW has been investigated mainly within the context of sepsis and septic shock, and it seems to be associated with the severity of respiratory dysfunction and mortality [2,4,5,7,15-17]. However, ALI and ARDS may also occur in patients without sepsis. Thus it is relevant to study EVLW in larger populations at high risk of developing the disease. These populations would encompass critically ill patients with systemic inflammation due to any cause (septic and nonseptic) and shock. It is also unclear which EVLW index is the most useful measure. Most reports regarding EVLW have used an index based on actual body weight (ABW). Three recent studies indicate that using predicted body weight (PBW) may be a better predictor of survival and disease severity [2-4]. Indexing EVLW to PBW instead of to ABW has been shown to improve the correlation between EVLW and LIS and the PaO_2_/FiO_2 _ratio [3]. EVLW indexed to pulmonary blood volume (PBV) is another measure and is thought to reflect increased hydrostatic pressure and pulmonary permeability [5-7,18]. It has been proposed as a useful index for differentiating the two mechanisms of increased EVLW [18].

These considerations led us to ask the following questions about critically ill patients with shock who are at risk for developing lung injury. (1) How well do different EVLW indices measure the severity of lung injury? (2) How well do the different EVLW indices relate to ICU mortality? (3) By applying EVLW as a bedside test, can the chances of diagnosing lung injury be increased? We investigated various indices of EVLW in relation to the presence and severity of lung injury and ICU mortality. Finally, we investigated the diagnostic value of the various indices for ALI, ARDS and severe lung injury (sLI) as defined by the NAECC criteria and LIS, respectively.

## Materials and methods

The present study was approved by the Regional Ethical Review Board, Lund, Sweden (Dnr.187/2005). Informed consent was sought either from the patient or, if not possible, from the patient's next of kin. The study design comprised a single-centre, prospective observational cohort of critically ill patients admitted to the mixed-bed ICU of Skåne University Hospital, Malmö, Sweden. Fifty-five consecutive patients with the systemic inflammatory response syndrome (SIRS) and shock despite fluid resuscitation were included. Specifically, patients were older than 18 years of age who met the SIRS criteria [19] and exhibited 'circulatory failure', defined as the failure to maintain mean arterial pressure ≥70 mmHg despite adequate fluid resuscitation according to the Surviving Sepsis Campaign algorithm [20]. Exclusion criteria were pregnancy, abnormalities of coagulation, fibrinolytic therapy, compromised immunity or a Do Not Attempt Resuscitation order. Patients could be included only once.

'Sepsis' was defined according to the criteria published by Bernard *et al. *[21]. ALI and ARDS were defined by the criteria set forth by the NAECC [22]. sLI was defined using the LIS proposed by Murray *et al. *[23], with sLI indicated by a score > 2.5. Acute Physiology and Chronic Health Evaluation II (APACHE II) scores [24] were calculated at admission, and Sequential Organ Failure Assessment scores [25] were calculated on each day of the study period. Ventilator settings (Evita XL ventilator; Dräger, Lübeck, Germany), including positive end-expiratory pressure (PEEP) and FiO_2_, were recorded, and if the patient was not mechanically ventilated, FiO_2 _was obtained from conversion according to commonly used tables [26]. An arterial blood sample was obtained every 6 hours. A bedside chest X-ray (CXR) was obtained at the time of inclusion and thereafter at the treating physician's discretion. X-rays were analysed for quadrants of alveolar consolidation (CXR score) as part of the LIS calculation [23].

All patients were initially treated according to international guidelines for the management of sepsis and septic shock [20]. This set of guidelines was applied to all patients at study inclusion because we were not able to identify at the outset all patients with sepsis. After the initial resuscitation period, fluids were given at the treating clinician's discretion. Regardless of shock aetiology, ventilator settings were set at 6 to 8 ml/kg PBW. Permissive hypercapnia was accepted. PEEP was adjusted to maximise compliance and oxygenation using a decremental PEEP trial. Recruitment was performed at the clinician's discretion. Patients were monitored according to standard ICU routines but also were treated with a 5-French femoral artery catheter (PV2015L20N; PULSION Medical Systems, Munich, Germany) and, if not already existing, a central venous catheter inserted into the internal jugular or subclavian vein.

PiCCO calibration and analysis were performed within 6 hours of study inclusion using mean values from three 20-ml iced saline injections. The method is based on measurement of temperature change over time in the femoral catheter after injection of cold saline solution into the central venous catheter. The transpulmonary thermodilution curve obtained is then analysed to calculate the cardiac output using the Stewart-Hamilton algorithm. Intrathoracic thermal volume and the pulmonary thermal volume are derived from the mean transit time and the exponential downslope time of the thermodilution curve. On the basis of these data, volumetric variables, including EVLW, may be estimated; their derivation has been described in detail previously [1,14-16]. Measurements taken within the first 6 hours of study inclusion made up the data set for this study.

EVLW was indexed to ABW, PBW and PBV. PBW (kg) was calculated as 50 + 0.91 for males (height = 152.4 cm) and 45.5 + 0.91 for females (height = 152.4 cm). We studied these EVLW indices within 6 hours of study inclusion. The relationship between EVLW indices and respiratory parameters (presence of ALI and ARDS, sLI, PaO_2_/FiO_2_, CXR score and PEEP) to ICU mortality were examined.

### Statistical analysis

Sample size was powered to detect a minimum difference between survivors and nonsurvivors of 2 ml/kg EVLW with a 2 ml/kg standard deviation of residuals, α = 0.05 and β = 0.8 using a *t*-test. These data gave us a sample size of 17 patients; however, because we were unsure of the variability of the data, and based on sample sizes in previous studies, we tripled our sample size. Data are presented as medians [IQR]. For correlations between two variables, Spearman's rank-correlation test was used; for differences between two groups, the Mann-Whitney *U *test was used. For comparison of multiple groups, analysis of variance on ranks was used and a Bonferroni correction was applied. Testing of proportions was carried out using Fisher's exact test. Significance was set at *P *< 0.05. Normality was tested for using the Kolmogorov-Smirnov test. The analyses were performed using SPSS version 16.0 software (SPSS Inc, Chicago, IL, USA) and SigmaStat version 3.5 for Windows software (Systat Software, Inc, San Jose, CA, USA).

For the evaluation of the diagnostic accuracy of each EVLW index, we calculated the positive likelihood ratio (LR+) and negative likelihood ratio (LR-), where LR+ is the sensitivity/(1 - specificity) and LR- is (1 - sensitivity)/specificity. The pretest odds of disease is given by *P*/(1 - *P*), where *P *is the probability of the disease in the current population. The posttest odds given a positive test are the product of the LR+ and pretest odds, whereas the posttest odds given a negative test is the product of the LR- and the pretest odds.

## Results

The original study included 55 consecutive patients. Two were excluded because of their lack of consent. Two other patients never received a femoral catheter because of technical difficulties (one with morbid obesity and one who had undergone massive aortofemoral surgery) and were excluded from further analysis. The remaining 51 patients presented no major technical difficulties and experienced no significant adverse events. At the time of inclusion, we managed to obtain EVLW data from 86% of the patients, and after 6 hours we had taken at least one measurement from all included patients. Thirty-four patients (67%) had septic shock according to the predefined criteria [21]. The remaining 17 patients had shock due to other causes, including pancreatitis (5 patients), post-noncardiac major surgery (5 patients), intoxication and multiorgan failure (2 patients) and gastrointestinal bleeding and portal hypertension (1 patient). In four patients, the cause of shock and organ failure was never established, although sepsis could not be ruled out. The patients' characteristics and clinical parameters are shown in Table 1.

**Table 1:** Characteristics of the study population

Patient characteristics	Data
Patients (*N*)	51
Gender (M/F)	35/16
Age at time of inclusion (years)	66 [57 to 76]
BMI (kg/m^2^)	25.8 [23.4 to 28.9]
Proportion with sepsis (%)	67
ICU mortality (%)	29
6-month mortality (%)	37
Proportion with ALI (%)^a^	35
Proportion with ARDS (%)^a^	29
Proportion with sLI (%)^b^	18
APACHE II score	24 [19 to 29]
SOFA score	12 [9 to 14]
PaO_2_/FiO_2 _ratio	230 [160 to 290]
PEEP (mmHg)	7 [5 to 10]
Arterial blood lactate (mmol/L)	3.0 [1.9 to 4.5]
CI (L/min/m^2^)	3.5 [2.8 to 4.5]
ITBVI (ml/m^2^)	1,010 [840 to 1,200]
EVLW/PBW ratio (ml/kg)	9.7 [7.7 to 12.4]
EVLW/ABW ratio (ml/kg)	8.3 [6.3 to 10.6]
EVLW/PBV ratio	1.8 [1.4 to 2.2]

ABW: actual body weight; ALI: acute lung injury; APACHE II: Acute Physiology and Chronic Health Evaluation II; ARDS: acute respiratory distress syndrome; BMI: body mass index; CI: cardiac index; EVLW: extravascular lung water; FiO_2_: fraction of inspired oxygen; ITBVI: intrathoracic blood volume index; PaO_2_: partial pressure of oxygen in arterial blood; PBV: pulmonary blood volume; PBW: predicted body weight; PEEP: positive end-expiratory pressure; sLI: severe lung injury; SOFA: Sequential Organ Failure Assessment. ^a^Defined by the NAECC [22]; ^b^defined by Murray's Lung Injury Score [23]. Data are medians [IQR].

### Extravascular lung water index and respiratory function

Eighteen (35%) and fifteen (29%) of the fifty-one patients fulfilled the NAECC criteria for ALI and ARDS, respectively. In contrast, only nine patients (18%) patients fulfilled the criteria for sLI according to Murray's LIS. The different EVLW indices were modestly correlated with PaO_2_/FiO_2 _(*r *= -0.371 to -0.487, *P *= 0.001 to 0.007) and CXR score (*r *= 0.255 to 0.455, *P *= 0.002 to 0.09), but not with PEEP.

Patients with increased EVLW indexed to body weight [> 10 ml/kg] had significantly lower oxygenation than those with normal EVLW. For EVLW/ABW, the data were 149 [111 to 234] vs 246 [192 to 301], *P *= 0.006; and for EVLW/PBW, the data were 158 [121 to 241] vs 256 [198 to 302], *P *= 0.004. Similar results were obtained for EVLW/PBV: 193 [143 to 282] vs 270 [220 to 289], *P *= 0.03. EVLW indexed to ABW and PBW were significantly higher in patients with ALI and ARDS (Figures 1a and 1b). EVLW indexed to PBV was also higher in these patients (Figures 2a and 2b). There were significant incremental increases in EVLW indices with each increasing stratum of the LIS score (Figure 3).

**Figure 1:** **Extravascular lung water indexed to actual and predicted body weight in patients with or without acute lung injury and/or acute respiratory distress syndrome**. **(a) **Extravascular lung water (EVLW) indexed to actual body weight (ABW) and predicted body weight (PBW) in patients with or without acute lung injury (ALI). Filled boxes = patients with ALI, unfilled boxes = patients without ALI (ABW: 10.4 [7.4 to 16.7] vs 7.8 [5.9 to 9.6], *P *= 0.01; PBW: 12.4 [9.4 to 17.7] vs 8.2 [7.5 to 10.9], *P *= 0.01). **(b) **EVLW indexed to ABW and PBW in patients with or without ARDS. Filled boxes = patients with ARDS, unfilled boxes = patients without ARDS (ABW: 10.0 [8.4 to 16.7] vs 7.8 [5.9 to 9.6], *P *= 0.01; PBW: 12.4 [9.4 to 17.7] vs 8.3 [7.5 to 10.9], *P *= 0.01). Data are medians [IQR]. *P < 0.05.

**Figure 2:** **Extravascular lung water indexed to pulmonary blood volume in patients with or without acute lung injury and/or acute respiratory distress syndrome**. **(a) **Extravascular lung water (EVLW) indexed to pulmonary blood volume (PBV) in patients with or without acute lung injury (ALI). Filled boxes = patients with ALI, unfilled boxes = patients without ALI (PBV: 2.1 [1.6 to 3.0] vs 1.6 [1.3 to 1.9], *P *= 0.02). **(b) **EVLW indexed to PBV in patients with or without acute respiratory distress syndrome (ARDS). Filled boxes = patients with ARDS, unfilled boxes = patients without ARDS (2.3 [1.6 to 3.1] vs 1.7 [1.3 to 1.9], *P *= 0.04). Data are medians [IQR]. *P < 0.05.

**Figure 3:** **Boxplots for extravascular lung water stratified by Lung Injury Score**. *P < 0.05 and **P < 0.01. Because there were only two patients in the group with Lung Injury Score (LIS) > 3, the group was omitted from statistical analyses and data are not shown. ABW: actual body weight; EVLW: extravascular lung water; PBV: pulmonary blood volume; PBW: predicted body weight.

### Extravascular lung water and mortality

All three EVLW indices were significantly higher in nonsurvivors vs nonsurvivors, respectively: EVLW/ABW 7.4 [5.9 to 9.4] vs 9.1 [7.9 to 12.9], *P *= 0.02; EVLW/PBW 9.1 [7.2 to 11.6] vs 10.6 [9.5 to 13.0], *P *= 0.05; EVLW/PBV 1.6 [1.3 to 2.0] vs 2.0 [1.6 to 2.6], *P *= 0.03 (Figure 4). The corresponding LR+ and LR- as well as pre- and posttest odds of death given a positive EVLW test are shown in Table 2.

**Figure 4:** **Extravascular lung water and mortality**. Filled bars = nonsurvivors, unfilled bars = survivors. *P < 0.05. ABW: actual body weight; EVLW: extravascular lung water; PBV: pulmonary blood volume; PBW: predicted body weight.

**Table 2:** Positive and negative likelihood ratios and pre- and posttest odds for mortality, given a positive extravascular lung water test

	EVLW alone				Combined with ALI				Combined with ARDS				Combined with sLI			
	
EVLW index	LR+	LR-	Pretest odds	Posttest odds	LR+	LR-	Pretest odds	Posttest odds	LR+	LR-	Pretest odds	Posttest odds	LR+	LR-	Pretest odds	Posttest odds
EVLW/ABW	1.83	0.55	0.38	0.69	2.27	0.70	0.38	0.86	1.89	0.79	0.38	0.71	4.40	0.70	0.38	1.66
EVLW/PBW	1.41	0.72	0.38	0.53	1.51	0.88	0.38	0.57	1.76	0.85	0.38	0.67	1.98	0.88	0.38	0.75
EVLW/PBV	2.11	0.59	0.38	0.80	1.76	0.85	0.38	0.67	2.11	0.86	0.38	0.80	3.52	0.78	0.38	1.33

ABW: actual body weight; ALI: acute lung injury; ARDS: acute respiratory distress syndrome; EVLW: extravascular lung water; LR-: negative likelihood ratio; LR+: positive likelihood ratio; PBV: pulmonary blood volume; PBW: predicted body weight; sLI: severe lung injury. A positive EVLW test was defined as EVLW/ABW ratio > 10 ml/kg, EVLW/PBW ratio > 10 ml/kg and EVLW/PBV ratio > 1.5.

### Diagnostic value of extravascular lung water

Depending on which index was used, EVLW identified between 44% and 100% of all patients with sLI (LIS > 2.5), 27% to 33% of those with ALI and 33% to 38% of those with ARDS. The sensitivities, specificities, LR+ and LR- and pre- and posttest odds for making a diagnosis of ALI, ARDS or sLI using various EVLW indices are shown in Table 3. By applying EVLW measurement as a bedside test, the posttest OR for the diagnosis of ALI and ARDS increased more than threefold when EVLW/ABW was used (from 0.55 to 1.8 for ALI, from 0.42 to 1.33 for ARDS). When using the same index, the posttest OR for sLI increased twofold.

**Table 3:** Sensitivity, specificity and positive and negative likelihood ratios of EVLW/ABW, EVLW/PBW and EVLW/PBV for diagnosis of acute lung injury, acute respiratory distress syndrome or severe lung injury

EVLW index	ALI	ARDS	sLI
EVLW/ABW			
Sensitivity	0.50	0.53	0.44
Specificity	0.85	0.83	0.76
LR+	3.30	3.2	1.87
LR-	0.60	0.56	0.73
Pretest odds	0.55	0.42	0.21
Posttest odds +	1.80	1.33	0.40
Posttest odds -	0.32	0.23	0.16
EVLW/PBW			
Sensitivity	0.61	0.60	0.67
Specificity	0.70	0.67	0.81
LR+	2.02	1.80	3.50
LR-	0.56	0.60	0.41
Pretest odds	0.56	0.42	0.21
Posttest odds +	1.10	0.75	0.75
Posttest odds -	0.30	0.25	0.09
EVLW/PBV			
Sensitivity	0.89	0.87	1.0
Specificity	0.52	0.47	0.88
LR+	1.83	1.64	8.4
LR-	0.22	0.28	0
Pretest odds	0.55	0.42	0.21
Posttest odds +	1.00	0.68	1.79
Posttest odds -	0.12	0.12	0

ABW: actual body weight; ALI: acute lung injury; ARDS: acute respiratory distress syndrome; EVLW: extravascular lung water; LR-: negative likelihood ratio; LR+: positive likelihood ratio; PBV: pulmonary blood volume; PBW: predicted body weight; sLI: severe lung injury. Posttest odds given a positive (posttest odds +) or negative EVLW test (posttest odds -) are also shown. Positive EVLW tests were defined as EVLW/ABW > 10 ml/kg, EVLW/PBW > 10 ml/kg and EVLW/PBV > 1.5.

In comparison, using EVLW/PBV as a bedside test increased the posttest OR for ALI and ARDS by 1.8 and 1.6 times, respectively, whereas the posttest OR for sLI increased more than eightfold. The posttest OR for lung injury by any definition decreased markedly given a negative EVLW test.

## Discussion

Our main finding is that increased EVLW adds diagnostic value in identifying patients with lung injury. Furthermore, it was significantly associated with disease severity and mortality. These findings support previous studies in which EVLW was found to be useful in characterising the severity of respiratory disease in patients with sepsis and those with ARDS [2-5,15-18,27]. We have shown in the present study that measurement of EVLW early during ICU admission in a wider population of critically ill patients at risk of developing lung injury is of both diagnostic and clinical significance. This was seen for all EVLW indices.

As a bedside test, EVLW/PBV provided excellent diagnostic accuracy for identifying patients with sLI according to Murray's LIS. For the diagnosis of ALI and ARDS, EVLW/ABW performed best as demonstrated by higher LR+. The application of increased EVLW as a bedside test improved the diagnostic accuracy for ALI, ARDS and sLI with two- to eightfold increases in the posttest OR observed in this population. Importantly, a negative EVLW test markedly decreases the OR of lung injury diagnosis, thus helping to rule out disease [28].

'Ruling in' disease may not translate to real clinical outcomes, hence there is a need to further assess the utility of EVLW in these terms. The present study shows not only that EVLW measured early during ICU admission may be used as a marker of respiratory dysfunction in patients with shock but also that EVLW is increased in nonsurvivors. This is consistent with earlier studies of patients with sepsis and ARDS [2-5,15-18] and extends current knowledge by showing that the posttest OR for mortality increases when EVLW is used as a diagnostic test, making this test clinically relevant. This is particularly true when combined with a prior diagnosis of ALI, ARDS or sLI, where the odds of mortality increase even further. The clear relationship between EVLW and several indicators of respiratory function, as well as the mortality seen in this study, support the utility of this bedside index for improved diagnosis and risk stratification early during ICU admission.

Theoretically, PBW seems to be a more logical index than ABW because lung volume does not increase with body fat. Because many critically ill patients are overweight [29], EVLW/PBW should be a better index. Although we found significant correlations between EVLW/PBW and respiratory function, EVLW/PBW demonstrated a weaker statistical relationship to mortality than EVLW/ABW or PBV. These results are in contrast to previous findings that indexing with PBW improved disease characterisation and correlations with survival [2-4]. One explanation for this discrepancy is that our patient population was not grossly overweight, with a median body mass index (BMI) of 25.8 kg/m^2^. Furthermore, there were significant differences in BMI between survivors and nonsurvivors, with the latter having lower BMI values, hence confounding any possible effect of adjustment for overweight. This study was conducted in a heterogeneous population at risk for developing lung injury, whereas researchers in previous studies investigated populations with established ARDS [2-4].

Another potentially attractive index to use is EVLW/PBV [6,7,18]. This index differs from EVLW adjusted for body weight in that it is thought to reflect increased lung water due to excessive hydrostatic pressure and vascular permeability independently of fluid status [6,7]. A recent study suggested that EVLW/PBV may even be useful for differentiating hydrostatic and pulmonary permeability mechanisms of increased EVLW [18]. EVLW/PBV consistently produced the lowest LR- compared to the other indices, reinforcing its usefulness in ruling out disease [28]. When measured against the 'gold standard' of sLI using Murray's LIS, EVLW/PBV performed well as a diagnostic test, with excellent LR+ and LR- values. With regard to the posttest odds of mortality, EVLW/PBV did not perform better than EVLW/ABW.

How may these results be applied clinically? First, we believe that EVLW may be used as an adjunct in the characterisation of sLI. There has been much debate regarding the usefulness of the NAECC criteria and the lack of specificity of LIS and PaO_2_/FiO_2 _in predicting mortality, leading to a search for more 'objective' criteria for ARDS [11] and for assessing the severity of lung injury [8]. Although the present study is not the first to report a relationship between EVLW and mortality, we have shown by calculating the LR+ and posttest odds [28] that increased EVLW confers additional diagnostic value for the identification of patients with lung injury and raises the odds for mortality, thus supporting its clinical relevance. This is particularly true when combined with a diagnosis of ALI, ARDS or sLI. This relationship was present at an early stage (within 6 hours of study inclusion) and was the first to document a stepwise relationship with deteriorating lung function. Our study also shows that the findings regarding increased EVLW applies to a population with shock and not only in patients with confirmed sepsis and/or ARDS. Early and correct identification of sLI patients at high risk of death allows the application of different treatment strategies and facilitates the design of clinical trials based on more robust criteria, issues previously identified as important for future research [8].

Our study has a number of limitations. Because of its design, this study cannot definitively answer the question whether EVLW is a better diagnostic test than the NAECC and LIS criteria, because EVLW would have to be compared to a gold standard which does not, at present, exist. Although power calculations were based on previously available data, our sample size was relatively small. A larger study would have allowed us to conduct multivariate regression analysis to establish whether EVLW is an independent risk factor for mortality as described by Craig *et al. *[4]. Although we used a pragmatic definition of 'sepsis' [21], we cannot exclude that some of the patients in the non-septic shock group also in fact had sepsis. Furthermore, this group represents only a limited proportion of the study population and a larger number of patients may have influenced the results. The study was not designed to investigate possible pathophysiological differences between EVLW/PBV and EVLW indexed to body weight. There is a mathematical coupling between intrathoracic thermal and blood volumes on which EVLW calculation is dependent. These and unaccounted for heterogeneous changes in ventilation and perfusion may have influenced the results. We sought only to generate hypotheses in this prospective, observational study; therefore, we cannot provide mechanistic explanations regarding EVLW and its relationship to clinical outcomes. Studies evaluating the incremental value of adding EVLW to current diagnostic criteria for the prognosis of clinical outcomes would be a logical next step in future research.

## Conclusions

In this study of critically ill patients with systemic inflammation and shock, EVLW measured early during the course of disease was correlated with respiratory function. Using EVLW as a bedside test conferred added diagnostic value for the identification of patients with lung injury. Furthermore, increased EVLW was related to severity of lung disease and mortality, confirming the results of previous studies in patients with ALI/ARDS and sepsis. Combining increased EVLW and a diagnosis of ALI, ARDS or sLI increases the posttest odds of ICU mortality. EVLW/ABW and PBV demonstrated the best diagnostic performance in this population. Prospective studies evaluating the value of adding EVLW to current diagnostic criteria for the prognosis of clinical outcome in at-risk populations and as a basis for tailored interventions are logical proposals for future research.

## Key messages

◆ EVLW is significantly related to the severity of lung injury and mortality in patients with shock, regardless of which index is used.

◆ Increased EVLW provides additional diagnostic value for lung injury.

◆ Increased EVLW increases the odds of mortality, especially when combined with a diagnosis of ALI, ARDS and sLI.

◆ EVLW indexed to ABW and PBV provides the best diagnostic and prognostic information in this patient population.

## Abbreviations

ABW: actual body weight; ALI: acute lung injury; ARDS: acute respiratory distress syndrome; BMI: body mass index; CXR: chest X-ray; EVLW: extravascular lung water; LIS: Lung Injury Score; LR+: positive likelihood ratio; LR-: negative likelihood ratio; NAECC: North American-European Consensus Conference; PBV: pulmonary blood volume; PBW: predicted body weight; PEEP: positive end-expiratory pressure; posttest odds +: posttest odds of disease given positive test; posttest odds -: posttest odds of disease given negative test; SIRS: systemic inflammatory response syndrome; sLI: sLI.

## Competing interests

MC has received travel reimbursements from PULSION Medical Systems AG, Munich, Germany.

## Authors' contributions

MC conceived the study; participated in study design, data collection and statistical analysis; and drafted the manuscript. LI participated in data collection, statistical analysis, data interpretation and drafting of the manuscript. JD and AE participated in study design, data collection and manuscript revision. JU participated in data analysis and interpretation and manuscript revision. LB, JR, EÅ and ML participated in data acquisition and manuscript revision. All authors read and approved the final manuscript for publication.
